RETRACTED

# Analysis of the Development Level of Green Economy in Different Regions Based on the GA-BP Model

**DOI:** 10.1155/2022/1587896

**Published:** 2022-09-09

**Authors:** Yanping Pu, Yonghui Cai

**Affiliations:** School of Public Affairs, Chongqing University, Chongqing 400044, China

## Abstract

The low-carbon economy is a green development mode of modern social and economic development. In this paper, an evaluation model of the green economy development level based on GA-BP is constructed, and the related parameters and network structure of the two algorithms are designed and optimized. The test results show that the predicted value of GA-BP has a high degree of fit to the actual value, and the data fitting performance is good. The prediction results are in good agreement with the objective reality, which is helpful to put forward appropriate development modes and development path suggestions for the regional development of the low-carbon economy.

## 1. Introduction

The green economy is a new term in people's vision in recent years, which is generally considered a low-carbon economy development mode in this century. For all countries in the world, it contains many development opportunities; but at the same time, there are many challenges. Since 2010, the Chinese government has issued several policies and measures to determine the direction for the development of China's low-carbon economy and has formulated a national goal of reducing carbon emissions by 40–45% by 2021 [1]. China's central region is currently in a period of rapid economic development, and energy consumption is also growing. At the present stage, the energy supply in the region still mainly relies on coal combustion. However, due to the limited investment capacity and technology, the overall proportion of green energy such as solar energy, geothermal energy, and natural gas is still low [2]. In order to get rid of the above difficulties as soon as possible, how to grasp the development opportunities, reduce the adverse effects caused by high carbon emissions, and how to optimize the energy consumption structure and industrial structure in the province, and gradually embark on the road of green development, so as to make greater progress in the province, these are a series of issues to be considered.

As for the impact of different economic development stages, modes, and speeds on carbon emissions, as well as the evaluation indicators of low-carbon economic development, the research results are relatively rich. Most researchers use the extended input-output model, computable general equilibrium model, and comprehensive evaluation model to determine the low-carbon operation level [3]. A. S constructed a comprehensive evaluation model of a low-carbon economy, including economic growth, energy utilization, and carbon emissions, and used the model to evaluate carbon emissions in the UK [4]. Duarte explored the balance and market factors involved in the CGE model. It can simulate the relationship and role of various fields and departments, restore the economic situation more truly, and calculate the carbon consumption expenditure based on the cross-regional CGE model [5]. Based on his understanding of the low-carbon economy and energy composition, Wang determined that the core factor in the model was carbon intensity. He not only discussed the relationship between the two in an all-round way but also determined the indirect, direct, and overall effects of energy composition with the help of path analysis and obtained the specific action mechanism [6]. Zhang et al. evaluated the provincial low-carbon competitiveness by constructing the evaluation index system of low-carbon competitiveness, using the entropy method to give weight, and took Shaanxi Province as an example to study [7]. From the current research situation, the existing foreign achievements have opened up a new perspective on the aspects of carbon emission trading mechanism and driving force, low-carbon policy, and connotation. But there is a lack of analysis of the connotation of a low-carbon economy and related factors and mechanisms.

RETRACTED

In the measurement of green economy, the commonly used linear evaluation models such as multiple linear regression and stepwise regression cannot fully explain the relationship between carbon emissions and economic growth, and there is a correlation between the influencing factors, so it is difficult to be independent. In addition, the quantitative standards of qualitative indicators are not unified and there are great differences. As a result, the relevant research focus has shifted to the nonlinear model [8, 9]. Because of its algorithm characteristics, the back propagation neural network (BPNN) can possess self-learning and self-growth, so as to solve nonlinear problems, and with the advantage of a computer, it can deal with batch problems at the same time. The low-carbon development ability of the developed cities is evaluated by the grey relational model of low-carbon development [10]. Shi used the BPNN method to build the evaluation model of regional agricultural coordinated development under a low-carbon economy and used the panel data of regional agriculture in China as an example to conduct empirical research [11]. Fan selected regional GDP, population size, industrial structure, energy consumption of 10000 yuan GDP, and energy consumption structure as the influencing factors of carbon emissions, established the PSO-BP neural network model, and further forecasted the total amount and intensity of carbon emissions [12]. However, when using the BPNN to evaluate the level of economic development, it often falls into the dilemma of local minimum value and slow model learning. Because of its inherent global optimization ability and adaptive characteristics, the genetic algorithm (GA) has been used to optimize the BPNN. Aiming at the complex nonlinear relationship between regional economic development level and various influencing factors, Lu Ji added a genetic algorithm to the adjustment and optimization of weights and thresholds of the BPNN, and through simulation experiments, it was proved that the model established by the combination of the two had significant significance for the prediction of the real green economy [13].

RETRACTED

According to the above analysis, this paper introduces the BPNN optimized by GA into the evaluation of regional green economic development level and establishes a neural network model with a high fitting degree, so as to accurately analyze the carbon productivity, and based on the above analysis results, it puts forward appropriate development mode and development path suggestions for regional development of the low-carbon economy.

## 2. Evaluation System of Green Economy Development

### 2.1. Construction Principles

#### 2.1.1. Scientificity

The construction of the indicator system should adhere to scientific principles. All indicators can accurately explain the value of the low-carbon operation and can reflect the current low-carbon operation status and laws of various cities. Operability means that the selected indicators can correspond to accurate and reasonable data, which is conducive to induction and accounting. Meanwhile, the data which are difficult to select and quantify should be excluded. In this research, the experimental data are taken from the statistical yearbook of Hunan Province in 2020 and the statistical yearbook of various cities.

#### 2.1.2. Comprehensiveness

The indicator system should be comprehensive and targeted and should be able to explain the different levels involved in the low-carbon operation. At the same time, based on the specific situation of the province's low-carbon operation, the indicators that can reflect the actual situation and cover a wide range are selected to reduce the difficulty of operation.

#### 2.1.3. Regional Comparability

In practice, the qualitative principle should be strictly followed. The selected indicators can truly reflect the characteristics and evolution law of a low-carbon economy, and then, based on the quantitative principle, ensure that the indicators are easy to quantify and use quantitative data modeling to carry out the final evaluation. In view of the large differences in the land area, economic situation, and total population of each city, the scale of each index is relatively large, which can be expressed by per capita data as much as possible, so as to make a more reliable comparison among cities.

RETRACTED

### 2.2. Index Description

Based on the meaning of low-carbon economy, the criteria for the establishment of indicators, and the idea of creating indicators, this paper selects a total of 22 specific indexes that can represent five aspects in the indicator system of regional differences in low-carbon economic development, as shown in Figure 1.

Low-carbon production reflects the low-carbon situation of various urban production areas. It can be seen from the data on the high carbon emission ratio of the province that the key indicator of carbon production in the province is the low-carbon production ratio. The specific indicators include carbon productivity, energy consumption per unit GDP, and relevant indicators of the three industrial structures. Low-carbon consumption: this part involves energy utilization rate and consumption structure. The first index measures the per capita energy consumption capacity, which can be obtained by comparing the total energy consumption with the total population. The second index can be obtained by comparing the total carbon emissions with the total population.

The low-carbon technology is the basic technical support for low-carbon operations in various regions. The relevant indicators include the ratio of R&D funds to GDP, and the larger the R&D investment amount, the more attention is paid to science and technology and technological change. The other two indexes are positive, reflecting the management level of toxic waste in urban life and industry.

Low-carbon environment presents the carbon sink of each city. With the help of this index, we can know the current local greening situation and environmental conditions. The last index is the proportion of the total area of local green space in the total area of the city, which is a key indicator to reflect the urban environment and social welfare.

In terms of a low-carbon society, the larger the corresponding value, the stronger the obstacle to local low-carbon operation. Except for these two indexes, the rest are positive indicators.

## 3. Evaluation Model of Green Economy Development Level Based on GA-BP

### 3.1. BP Design

In this paper, the number of nodes in the input layer, hidden layer, and output layer is mainly solved when the BPNN model is designed, as well as the number of hidden layers and related structural parameters.

RETRACTED

#### 3.1.1. Number of Nodes in Layers

The number of nodes in different layers is usually determined by the independent variable and dependent variable extracted from the modeling of practical problems. In the evaluation model of the green economic development level studied in this paper, the index influencing the development level of the green economy is taken as input variables to enter the BP terminal. According to the evaluation index screening and optimization results in Chapter 2, the number of BP input layer nodes is 22. The purpose of the study is to obtain a green economy development level, so the number of nodes in the output layer is 1.

(1) $$\begin{array}{c} q=\sqrt{n+m}+\alpha . \end{array}$$

According to formula (1), the number of hidden layer nodes ranges from 4 to 13. In the process of model debugging, on the premise of consistent training sample data, the global error of neural networks with different numbers of hidden layer nodes can be measured, respectively, and a reasonable number of nodes can be finally determined. In this paper, first, the appropriate range of nodes is determined according to the empirical formula, and then, the optimal number of nodes is found by the trial and error method.

#### 3.1.2. Hidden Layer Number

The structure design of the BPNN is very important and complex, and the complex points focus on the determination of the number of hidden layers. At present, there is no scientific method to confirm, but according to Kolmogorov theorem, a basic BPNN (1 input layer, 1 hidden layer, and 1 output layer) can approach any nonlinear continuous function with arbitrary precision as long as the number of nodes in the hidden layer can be changed. In other words, a three-layer BPNN can theoretically solve any nonlinear problem. Moreover, although increasing the number of hidden layers will reduce the probability of the model falling into the local minimum, it will make the network structure more complex and may reduce the convergence speed of the model. Therefore, it is necessary to be cautious in increasing the number of hidden layers. According to the actual evaluation model of green economic development level, the BPNN with one hidden layer can better interpret the case data. Therefore, the number of hidden layers is set to 1.

#### 3.1.3. Related Parameters

The initial weight is equivalent to a starting line for the BPNN. If the training result is more accurate, the training result will be more accurate. Generally speaking, the initial weight is set between 0 and 1, which is randomly generated by the computer. However, in the actual problem solving, training the network with different weights will lead to the convergence of different local extremum each time. Based on this, this paper proposes to introduce a genetic algorithm to find the optimal weight.

RETRACTED

The learning rate will affect the weight increment of single-cycle training. Too high, a learning rate will destroy the stability of the model, and too low, a learning rate will lead to a great increase in training time. In general modeling, the range of learning rate is 0.01–0.8. In order to ensure the stability of the model, researchers tend to use a smaller learning rate. In this paper, the learning rate of BPNN is set to 0.1.

The training error can be set to different values due to the different expectations of the designer. Generally speaking, when the accuracy requirement of the problem is high, it is necessary to set a small training error. In this paper, the expected error of BPNN is set as 0.00001.

### 3.2. GA Design

In this paper, we mainly solve the problems of the coding method, fitness function, genetic manipulation, and parameter control.

#### 3.2.1. Fitness Function

Different from other optimization algorithms, the genetic algorithm only uses the fitness function as the basis to find the optimal value. However, the constraint of the fitness function is very loose, and only need not be negative. In actual problem-solving, the appropriate fitness function is selected according to the different requirements of specific problems. When designing the fitness function of the genetic algorithm, based on the global error *E* of the BPNN, the weight coefficient method is used to construct the fitness function:

(2) $$\begin{array}{c} \text{Fun}=\sum_{i=1}^{N}a_{i}\cdot E_{p}+a\cdot E, \end{array}$$

where *a*_*i*_ is the proportion of each sample error in the fitness function of the BPNN; *a* is the proportion of all sample errors in the fitness function of the BPNN.

#### 3.2.2. Genetic Manipulation

Selection: in this paper, the fitness ratio method is used in this operation. This method is the most commonly used selection operation to construct genetic algorithm-related models. The probability is proportional to the fitness of each individual. If the population size is P and the fitness value of individuals is *f*, then the calculation of selection probability is as follows:

(3) $$\begin{array}{c} P=\frac{f_{i}}{\sum_{i=1}^{P}f_{i}}. \end{array}$$

The method is in line with the law of biological evolution: the better an individual is, the greater the probability that it will be passed on.

Crossover: in the crossover operation of the genetic algorithm, the codes at any position of the chromosome will be exchanged with a set probability. In this paper, a single-point crossover is used, that is, a crossover point is randomly set in the chromosome string of an individual. When the crossover operation occurs, some structures of the two individuals before or after the crossover point are exchanged to generate a new individual. In general, the range of cross probability is 0.4–0.9. In this paper, based on the stability of the model structure, the cross probability is set as 0.4.

RETRACTED

Variation: it refers to the inversion of the selected chromosome coding value, i.e., 1 ⟶0 or 0⟶1. The main steps of mutation operation are as follows: the chromosome positions are randomly determined in the coding set of all individuals in the population, and then, the chromosomes of these chromosome positions are mutated according to the preset mutation probability.

Among them, mutation probability is an important parameter, whether the algorithm can quickly and accurately converge to the optimal solution which is directly affected by it. The larger mutation probability will make the genetic algorithm generate new individuals, expand the solution space, and deal with more variety of changes, but at the same time, it will reduce the convergence speed of the algorithm. In general, the mutation probability is between 0.001 and 0.01 and usually takes a smaller value. In this paper, the mutation probability of the genetic algorithm is set as 0.001.

#### 3.2.3. Population Size

Therefore, the larger the number of global solutions, the greater the number of solutions. However, if the population size is too large, the amount of calculation will be greatly increased. In this paper, by substituting different size populations into the genetic algorithm and considering the accuracy and training time of the algorithm, an optimal value is determined.

#### 3.2.4. Iterations

The training times of the whole model before the algorithm stops running. Currently, there is no suitable method or conclusion to determine the number of iterations. It is generally believed that the optimal solution is obtained when the optimal individuals obtained by the algorithm do not change anymore. At this time, increasing the number of iterations has little effect on the algorithm results. In this paper, the genetic algorithm iteration number setting method is consistent with the method of determining the population size. Through repeated experiments, the optimal iteration number is determined to be 50.

## 4. Model Training and Simulation

### 4.1. Data Input

This paper extracts the data of 31 regions in China from 2014 to 2020, carries out principal component analysis, reduces the data redundancy of the evaluation system, selects the important principal components whose cumulative contribution rate reaches 85%, and takes their scores as the comprehensive evaluation samples. 80 samples were randomly selected from 100 samples as a training set, and the specific index data and housing price after quantification were put into the GA-BP model. The remaining 20 samples were tested for the accuracy and validity of the model after training.

RETRACTED

## 5. Results and Discussion

### 5.1. Model  Optimization

In the BPNN model, the number of hidden layer nodes is determined to be between 4 and 13 according to the empirical formula, and different node numbers are substituted into the model for training, as shown in Figure 2.

Figure 2 shows the mean data that the optimal number of nodes is determined to be 5. In this paper, optimal population size is determined by comparing the optimization accuracy and training time of the model under different groups. After many experiments, the test results of different population sizes as shown in Figure 3 are obtained.

The population size set in the genetic algorithm is determined as 10. The optimal fitness optimization process curve of GA is shown in Figure 4.

When the number of iterations reaches 50, the curve starts to be stable, which means that the model has converged, that is, the optimal value is found. Moreover, the running time of the model is shorter when the number of iterations is 50.

### 5.2. Regional Clustering Results

According to the optimal individual value of GA, the result of mapping high-dimensional data into two-dimensional space is obtained, as shown in Figure 5.

The number of 32 provinces and cities in China is ranked according to the country's GDP in 2021. For reasons of length, they are not listed. According to the cluster analysis of each sample, the economic development level of different regions can be roughly divided into four categories:

Category A (developed areas of green economy developed areas): Beijing and Shanghai; Category B (good developed areas of green economy): Tianjin, Zhejiang, Guangdong, Jiangsu, Fujian, Liaoning, Shandong, and Inner Mongolia; Category C (moderately developed areas of green economy): Chongqing, Hainan, Jilin, Hubei, Hebei, Shaanxi, Heilongjiang, Shanxi, Hunan, Ningxia, Jiangxi, Anhui, Sichuan, Henan, Xinjiang, and Guangxi; Category D (underdeveloped areas of green economy): Qinghai, Yunnan, Tibet, and Gansu, Guizhou. Among them, the development level of the green economy in Beijing and Shanghai is significantly higher than that in other regions. The economic development level of Guangdong, Zhejiang, Jiangsu, and Tianjin is also relatively high.

The influence factors of the economic system are complex, and the nonlinear characteristics of data are obvious. The genetic clustering algorithm is used to cluster the coordinated development level of the regional economy in China, which provides an intelligent method for regional economic analysis. Compared with the traditional clustering method, GA reduces the artificial selection factors and is more objective in classifying the development level of the green economy in China.

RETRACTED

### 5.3. Analysis of Model Prediction Results

After the optimization and adjustment of BP and GA parameters, the sample data are put into the model. After the optimal initial weights and thresholds are assigned to the BPNN, the prediction output, prediction error, and error percentage are obtained by training with sample data, as shown in Figure 6.

The fitting degree of BP-GA is better than that of actual data. According to the results of cluster analysis and prediction analysis, there is a big gap in the coordinated development level of the green economy among regions in China, and the level of the eastern region is higher than that of other regions. The gap between the Central and Western regions has narrowed. The level of Northeast China has been improved; Tibet has developed rapidly due to the coordinated development of state support policies. Comprehensive analysis shows that it is a long-term task to coordinate the development of the green economy.

## 6. Conclusion

This paper uses GA to cluster and forecast the development level of the green economy. By constructing the evaluation system of green economy development, the GA-BP model is used to predict the development level of the regional green economy. The simulation results show that GA can realize data clustering analysis well. The prediction value of GA-BP has a high fitting degree with the actual value, the data fitting performance is good, and the prediction result is consistent with the objective reality. From the results of cluster analysis and prediction analysis, there is a big gap in the development level of the green economy in different regions of China, so it is a long-term task to coordinate the development of the green economy.

## Figures and Tables

**Figure 1:** The index system of regional differences in green economic development.

**Figure 2:** Training results of the BPNN model with different node numbers.

**Figure 3:** Test results of different population sizes.

**Figure 4:** GA optimal fitness optimization process.

**Figure 5:** Two-dimensional spatial mapping results of green economic development level in different regions.

**Figure 6:** Prediction output of the GA-BP model.

## Data Availability

The data used to support the findings of this study are available from the corresponding author upon request.
